The article "Long non‐coding RNA MEG3 silencing and microRNA‐214 restoration elevate osteoprotegerin expression to ameliorate osteoporosis by limiting TXNIP" was retracted in 2022. Reasons: signs of a paper mill; unreliable results or conclusions.

# Long non‐coding RNA MEG3 silencing and microRNA‐214 restoration elevate osteoprotegerin expression to ameliorate osteoporosis by limiting TXNIP

**DOI:** 10.1111/jcmm.16096

**Published:** 2021-01-03

**Authors:** ChangSheng Yang, ZhengTao Gu, Rui Ding, CaiQiang Huang, QingChu Li, DengHui Xie, RongKai Zhang, YiYan Qiu

**Affiliations:** ^1^ Division of Spine Surgery, Section II Department of Orthopedics The Third Affiliated Hospital of Southern Medical University Guangdong Provincial Key Laboratory of Bone and Joint Degeneration Diseases Southern Medical University Academy of Orthopedics of Guangdong Province Guangzhou China; ^2^ Department of Treatment Center For Traumatic Injuries The Third Affifiliated Hospital of Southern Medical University Guangdong Provincial Key Laboratory of Bone and Joint Degeneration Diseases Southern Medical University Academy of Orthopedics of Guangdong Province Guangzhou China; ^3^ Division of Joint Surgery Department of Orthopedics The Third Affiliated Hospital of Southern Medical University Guangdong Provincial Key Laboratory of Bone and Joint Degeneration Diseases Southern Medical University Academy of Orthopedics of Guangdong Province Guangzhou China

**Keywords:** differentiation, long non‐coding RNA maternally expressed gene 3, microRNA‐214, osteoblasts, osteoporosis, osteoprotegerin, proliferation, thioredoxin‐interacting protein

## Abstract

Studies have shown that long non‐coding RNA (lncRNA) MEG3 plays a key role in osteoporosis (OP), but its regulatory mechanism is somewhat incompletely clear. Here, we intend to probe into the mechanism of MEG3 on OP development by modulating microRNA‐214 (miR‐214) and thioredoxin‐interacting protein (TXNIP). Rat models of OP were established. MEG3, miR‐214 and TXNIP mRNA expression in rat femoral tissues were detected, along with TXNIP, OPG and RANKL protein expression. BMD, BV/TV, Tb.N and Tb.Th in tissue samples were measured. Ca, P and ALP contents in rat serum were also determined. Primary osteoblasts were isolated and cultured. Viability, COL‐I, COL‐II and COL‐Χ mRNA expression, PCNA, cyclin D1, OCN, RUNX2 and osteolix protein expresion, ALP content and activity, and mineralized nodule area of rat osteoblasts were further detected. Dual‐luciferase reporter gene and RNA‐pull down assays verified the targeting relationship between MEG3, miR‐214 and TXNIP. MEG3 and TXNIP were up‐regulated while miR‐214 was down‐regulated in femoral tissues of OP rats. MEG3 silencing and miR‐214 overexpression increased BMD, BV/TV, Tb.N, Tb.Th, trabecular bone area, collagen area and OPG expression, and down‐regulated RANKL of femoral tissues in OP rats. MEG3 silencing and miR‐214 overexpression elevated Ca and P and reduced ALP in OP rat serum, elevated osteoblast viability, differentiation ability, COL‐I and COL‐Χ expression and ALP activity, and reduced COL‐II expression of osteoblasts. MEG3 specifically bound to miR‐214 to regulate TXNIP. MEG3 silencing and miR‐214 overexpression promote proliferation and differentiation of osteoblasts in OP by down‐regulating TXNIP, which further improves OP.

## 1 INTRODUCTION

Osteoporosis (OP) refers to a systemic disease of bone structures giving rise to low bone mass reduction in bone mass caused by imbalance between bone formation and resorption ratio and the micro architectural deterioration, and it is also a severe health problem leading to great economic and social impacts.^1^ There are numerous factors which may account for the occurrence of OP, such as mechanical loading, heritable and non‐heritable factors, oestrogen deficiency during menopause and ageing caused by intracellular reactive oxidative species.^2^ In consideration of the stable rise in people's life expectancy and the substantial alterations in people's lifestyles in China in the past years, OP is likely to be more prevalent in the near future.^3^ Hence there is a pressing need for us to seek for more effective treatments for OP.

Long non‐coding RNAs (LncRNAs) refer to RNA transcripts (>200 nucleotides) with no or little protein‐coding ability which are capable of modulating gene expression via various mechanisms, such as mRNA splicing and epigenetic silencing.^4^ LncRNAs have been demonstrated to participate in OP. For example, a recent report has revealed that lncRNA CRNDE exerts effects on osteoclast proliferation through oestrogen deficiency in postmenopausal OP.^5^ Also, maternally expressed gene 3 (MEG3), an important lncRNA, has lately been proposed to depress osteogenic differentiation of bone marrow mesenchymal stem cells (BMSCs) in postmenopausal OP.^6^ There is a study showing that the binding relationship between microRNA (miR)‐214 and lncRNA MEG3.^7^ A prior literature has indicated the role of miR‐214 in primary OS via inhibiting osterix expression in bones.^8^ It has also been suggested that miR‐214 defends MC3T3‐E1 osteoblasts from H_2_O_2_‐induced apoptosis by restricting oxidative stress.^9^ Thioredoxin‐interacting protein (TXNIP) is a pervasively expressed protein which interacts and negatively modulates Thioredoxin expression and function.^10^, ^11^ Lekva T *et al* have proffered that TXNIP knockdown in osteoblasts boosts cell differentiation and osteocalcin (OCN) expression and secretion, and strengthens alkaline phosphatase (ALP) activity.^12^ Nicotinamide mononucleotide‐mediated repression of TXNIP/NLRP3 inflammasome pathway has been reported to attenuate aluminium‐induced bone loss.^13^ Nevertheless, little research has probed into the function of lncRNA MEG3 in OP. Therefore, we performed this study to figure out how MEG3 affects OP development by modulating miR‐214 and TXNIP.

## 2 MATERIALS AND METHODS

### 2.1 Ethics statement

Animals were treated humanely in compliance with the recommendations in the Guide for the Care and Use of Laboratory Animals of the National Institutes of Health. The protocol was approved by the Institutional Animal Care and Use Committee of The Third Affiliated Hospital of Southern Medical University, Guangdong Provincial Key Laboratory of Bone and Joint Degeneration Diseases, Southern Medical University, Academy of Orthopedics of Guangdong Province.

### 2.2 Experimental animals

Eighty female rats (3 months old, 226 ± 12 g) purchased from Guangdong Medical Laboratory Animal Center (Guangdong, China) were fed on standard feedstuff and kept in cages, free to feed and drink water (12‐hour day/night cycle, 23‐26°C, 40%‐70% relative humidity). An operation was performed after adaptive feeding in the laboratory.

### 2.3 Model establishment

Rats for OP modelling (n = 70) were intraperitoneally injected with 1% pentobarbital sodium (40 mg/kg). After completely anesthetized, the rats were fixed in the prone position to cut the clothing hair on the back. After the back skin was disinfected by iodine and alcohol, a longitudinal incision was made on both sides of the spine to separate the muscles and open the abdominal cavity. Then the left and right ovaries (carnation granules on the adipose tissue) were cut off, and the abdomen was sutured layer by layer with 2‐3 needles on both sides. After erythromycin eye ointment was applied to both eyes, the rats were put back into the cages in the prone position. The rats with sham operation (n = 10) were treated in the same way as above except that the uterus was not ligated and the ovaries were not removed.

### 2.4 Rat treatment

A week later, seventy successfully modelled rats were divided into 7 groups (n = 10) and respectively injected with si‐MEG3, si‐MEG3 negative control (NC), miR‐214 mimic, miR‐214 mimic NC, overexpressed (OE)‐MEG3 + miR‐214 mimic or OE‐MEG3 + miR‐214 mimic NC. At a week post modelling, all si‐MEG3/miR‐214 mimic/OE‐MEG3 and corresponding NC oligonucleotides or plasmids were subcutaneously injected once a week at 100 μL (5 μg oligonucleotide with transfection solution per rat). The sham‐operated rats were injected with the same amount of normal saline. At 4 w post‐injection, all rats were killed by cervical dislocation for subsequent indicator detection. siRNA targeting MEG3, miR‐214 mimic/inhibitor and MEG3 overexpression plasmid were all constructed and provided by GenePharma.

### 2.5 Detection of bone histomorphometric indicators

The femurs of all rats were fixed in periodate‐L‐lysine‐paraformaldehyde for 48 hours and then scanned on a CT machine according to relevant parameters. CTAn software was adopted to calculate bone mineral density (BMD), bone surface/bone volume (BS/BV), trabecular bone number (Tb.N) and trabecular thickness (Tb.Th).

### 2.6 Serum sample collection and determination of Ca, P and ALP levels

Before the rats were killed, blood was taken from the vein of posterior eyelid plexus, left for about 1 hour and centrifuged at 1358 × g at 4°C for 15 minutes to separate serum. The contents of Ca, P and ALP in blood were detected by an automatic biochemical analyser.

### 2.7 Bone tissue section preparation

After the muscle connective tissues surrounding 1/3 of the distal femur on the right side of rats were removed, the bone tissues were placed in 4% paraformaldehyde (pH 7.4, containing 0.1% diethyl pyrocarbonate) for 24 hours and decalcified in 10% ethylenediaminetetraacetic acid (EDTA) at 4°C for 8 weeks (EDTA was changed once every 4 to 5 days until the tissues became soft). Then, the tissues were immersed in 0.2 mol/L phosphate‐buffered saline (PBS) overnight, and separately soaked in 70%, 80%, 95% and absolute ethanol mixed with the same volume of n‐butyl alcohol for 1 hour, then permeabilized in xylene for 30 minutes, embedded in paraffin, finally sliced into 4‐μm sections along the longitudinal diameter of the femur and dried.

### 2.8 Haematoxylin and eosin (HE) staining and Masson staining

#### 2.8.1 HE staining

Tissue specimens were dewaxed with xylene, dehydrated with alcohol of descending concentrations, stained with haematoxylin solution for 5 minutes, then differentiated in acid water and ammonia water for 10 seconds, dehydrated in 70% and 90% alcohol for 10 minutes, and stained with alcohol eosin staining solution for 2‐3 minutes. The stained sections were subsequently dehydrated with absolute ethanol, permeabilized by xylene, sealed by Canadian gum with a cover slip, slightly dried and finally observed under the microscope.

#### 2.8.2 Masson staining

paraffin sections were deparaffinized and then chromized. Then the nucleus was stained with haematoxylin for 5‐10 minutes and with Masson ponceau acid fuchsin solution for 5‐10 minutes, differentiated with 1% phosphomolybdic acid solution for 3‐5 minutes, stained with aniline blue for 5 minutes, dehydrated with 95% and anhydrous alcohol, and finally observed under the microscope after xylene permeabilization and sealing with neutral gum.

### 2.9 Immunohistochemical staining

The prepared tissue sections were deplasticized, hydrated and put in 3% H_2_O_2_ for 10 minutes to block endogenous peroxidase, and placed into 0.01 mol/L citrate buffer (pH 6.0) for 5‐minutes antigen retrieval under high‐pressure steam. After cooled for 20 minutes, the sections were sealed with 5% goat serum for 20 minutes, supplemented with 40 μL goat anti‐osteoprotegerin (OPG) and receptor activator of nuclear factor кB ligand (RANKL) (both 1:150) polyclonal antibody, and placed in a wet box at 4°C overnight, followed by adding biotinylated rabbit anti‐goat immunoglobulin G secondary antibody (15 minutes) and horseradish peroxidase‐labelled streptavidin (15 minutes), and 3‐amino‐9‐ethylcarbazole staining under the microscope. At last, the sections were observed under the microscope after counterstained with haematoxylin and sealed with glycerine gelatin.

### 2.10 Isolation and culture of osteoblasts

On the ultra‐clean bench in the cell room, some cancellous bones of the femurs were cut into 2‐mm^3^ masses by a rongeur and other instruments, placed in a sterile 50 mL centrifuge tube, and then shaken repeatedly and rinsed 3 times with PBS until the cancellous bone granules became white honeycomb. Next, the samples were detached with 0.25% trypsin in an incubator at 37°C for 5 minutes, washed twice with α‐minimum Eagle's medium (α‐MEM) containing 10% foetal bovine serum (FBS), and rinsed once with PBS, then detached with 1 mg/mL type II collagen (COL‐II) at 37°C for 1.5 hours (shaken every 15 minutes), and then supplemented with α‐MEM containing 20% FBS to end the detachment. After centrifugation and 3 washes with α‐MEM containing 10% FBS (after each wash, bone tissues and cells were precipitated by centrifugation at 1000 r/min for 10 minutes), the samples were supplemented the culture solution (α‐MEM + 15% FBS + 100 U/mL penicillin + 100 μg/mL streptomycin) and triturated to free more osteoblasts. The cells were separately added 4 to 5 25‐cm^2^ cell culture flasks after trituration (some cells were separated and added to cell culture dish with a built‐in coverslip, and then VanGieson picric acid‐acid fuchsin staining, ALP staining, alizarin red staining (ARS) were performed for cell identification after the cells spread over the dish).

### 2.11 Osteoblast identification

After reaching confluence, the cells were detached with 0.25% trypsin‐EDTA solution and inoculated into a plate with a cover glass at 3 × 10^5^ cells/mL, and the osteoblast phenotype was identified as follows.

#### 2.11.1 VanGieson picric acid‐acid fuchsin staining

After confluence, the cells were fixed with 4% paraformaldehyde for 10 minutes, stained with Weigert iron haematoxylin dye solution for 5 minutes and VanGieson picric acid‐acid fuchsin staining solution for 5 minutes, and rapidly differentiated and dehydrated with 95% ethanol. Then the coverslip was placed under an inverted microscope for observation, and photographs were taken.

#### 2.11.2 ARS staining

After cell confluence for 8 d, the supernatant was removed, and cells were fixed with 95% ethanol for 2 minutes and air‐dried. Then, 2% alizarin red dye solution was prepared to stain the cells, and the staining reaction was terminated through 3 ddH_2_O washes. Then the cells were observed under a microscope, scanned and photographed after dried.

### 2.12 Cell transfection

The isolated OP osteoblasts were transfected with si‐MEG3, si‐MEG3 NC, miR‐214 mimic, miR‐214 mimic NC, miR‐214 inhibitor, inhibitor NC, OE‐MEG3 + miR‐214 mimic, or OE‐MEG3 + miR‐214 mimic NC, or not transfected with any sequence. Osteoblasts from sham‐operated rats were also used as a control.

#### 2.12.1 Transfection

Osteoblasts were seeded onto a sterile 6‐well culture plate. When the cells reached 30–50% confluence, si‐MEG3, si‐NC, miR‐214 mimic, mimic NC, miR‐214 inhibitor, Inhibitor NC, OE‐MEG3 + miR‐214 mimic and OE‐MEG3 + mimic NC transfected into osteoblasts cells. Transfection was performed using Lipofectamine 2000 from ThermoFisher Scientific (Waltham, MA, USA) according to the manufacturer's protocol.

#### 2.12.2 miRNA transfection efficiency

miR‐214 mimic/inhibitors were labelled with enhanced green fluorescent protein plasmid (pEGFP) (ELIM Biopharm, Hayward, USA). At 48‐hours post‐transfection with Lipofectamine 2000, the cell morphology was observed with an inverted fluorescence microscope GFP expression was tested in the same field and the number of cells with 5 green fluorescence and the total number of cells were counted. Transfection efficacy = number of green fluorescence cells/total number of cells.^14^ It was found that the transfection efficiency of Lipofectamine 2000 was 78% (Figure 1).

**Figure 1:** In the preliminary experiment, the green fluorescent protein reporter gene was utilzied to evaluate the efficiency of Lipofectamine 2000 and it was found that the transfection efficiency of Lipofectamine 2000 was about 78%. A, Cells were labelled by GFP; B, The transfection efficacy of miR‐214 mimic/inhibitor via Lipofectamine 2000

### 2.13 3‐(4,5‐dimethylthiazol‐2‐yl)‐2,5‐diphenyltetrazolium bromide (MTT) assay

Osteoblasts in each group were inoculated in a 96‐well cell culture plate at 1 × 10^5^ cells/mL and incubated for 24 hours. After cell attachment, the medium was substituted with 10% FBS and incubated with MTT solution (20 μL, 5 mg/mL) for 4 hours at 37°C. After removing the supernatant, 150 μL dimethyl sulphoxide was added to each well, shaken at low speed for 10 minutes and an microplate reader was adopted to detect the optical density (OD) value at 490 nm. Three independent replicate experiments were performed.

### 2.14 ALP staining with 5‐bromo‐4‐chloro‐3‐indolyl phosphate (BCIP)/nitrotetrazolium blue chloride (NBT) kits

Osteoblasts at passage 3 or in logarithmic phase were inoculated into a 6‐well plate at 1.0 × 10^5^ cells/well, and the medium was altered every 2 to 3 d. When the cell confluence was 60%, osteoblasts were fixed with 95% ethanol for 2 minutes and then dried. Then 2 mL BCIP/NBT staining working solution prepared at the reference ratio in the specifications (Nanjing Jiancheng Bioengineering Institute, Nanjing, China) was added add to be fully spread over the surface and incubated at 37°C in the dark for 30 minutes until the colour development was normal. After removing the BCIP/NBT staining working solution, the staining was ended by 1‐2 ddH_2_O washes, and the experimental results were recorded.

### 2.15 Reverse transcription quantitative polymerase chain reaction (RT‐qPCR)

Trizol (Invitrogen, Carlsbad, CA, ΜSA) method was adopted to extract total RNA from tissues and cells, and NanoDrop2000 (Thermo Fisher Scientific, Waltham, MA, USA) to determine the concentration and quality of RNA. RNA was reversely transcribed into cDNA according to the reverse transcription kit ReverTra Ace qPCR RT Kit (TOYOBO, Osaka, Japan) and stored at 4°C. RT‐PCR reaction system was prepared based on the Green kit (Takara, Dalian, China), and the primers were synthesized by BGI (Guangdong, China) (Table 1). U6 and glyceraldehyde‐3‐phosphate dehydrogenase (GAPDH) were the internal controls. The data were analysed by 2^‐ΔΔCt^ method. The experiment was repeated three times, and the data were averaged.

**Table 1:** Primer sequence

Gene	Primer sequence
MEG3	F: 5′‐ATCCGTCCACCTTGTCT‐3′
	R: 5′‐CCTCTTCATCCTTTGCCATC‐3′
miR‐214	F: 5′‐GACAGCAGGCACAGACA‐3′
	R: 5′‐GTGCAGGGTCCGAGG‐3′
TXNIP	F: 5′‐GAAGCTCCTCCCTGCTATATGGA‐3′
	R: 5′‐CCATGTCATCTAGCAGAGGAGTTGT‐3′
COL‐I	F: 5′‐TTTAATGGATAGGGACTTGTGTGAA‐3′
	R: 5′‐GAGAGAGAGAGAAGCTGAGGGTAGG‐3′
COL‐II	F: 5′‐CCCCATCTGCCCAACTGA‐3′
	R: 5′‐CTCCTTTCTGTCCCTTTGGT‐3′
COL‐X	F: 5′‐ACTTCTCTTACCACATACACG‐3′
	R: 5′‐CCAGGTAGCCCTTGATGATGTACT‐3′
U6	F: 5′‐ATTGGAACGATACAGAGAAGATT‐3′
	R: 5′‐GGAACGCTTCACGAATTTG‐3′
GAPDH	F: 5′‐ACGGCAAGTTCAACGGCACAG‐3′
	R: 5′‐GACGCCAGTAGACTCCACGACA‐3′

Abbreviations: COL, collagen; F, forward; GAPDH, glyceraldehyde‐3‐phosphate dehydrogenase; MEG3, maternally expressed gene 3; miR‐214, microRNA‐214; R, reverse; TXNIP, thioredoxin‐interacting protein.

### 2.16 Western blot analysis

Total protein of tissues and cells in each group were extracted, and protein concentration was measured with the bicinchoninic acid protein concentration determination kit (Beyotime Institute of Biotechnology, Shanghai, China). After the protein concentration in each group was adjusted to the same level, the extracted protein was added to the loading buffer and boiled at 95°C for 10 minutes, and each well was then loaded with 30 μg sample. Next, the protein was separated by 10% polyacrylamide gel electrophoresis (80 V for 30 minutes, then 120V), transformed to polyvinylidene fluoride (PVDF) membrane (300 mA, 60‐120 minutes) in ice water, and blocked in 5% bovine serum albumin for 2 hours. Primary antibody against TXNIP, proliferating cell nuclear antigen (PCNA), cyclin D1, OCN, runt‐related transcription factor 2 (RUNX2), Osteolix, OPG, RANKL (all 1:1000) and GAPDH (1:3000) (all from Abcam, Cambridge, MA, USA) were added and kept at 4°C overnight, and then, the corresponding diluted secondary antibody (MT‐BIO, Shanghai, China) was added and incubated for 2 hours, followed by development with chemiluminescent reagent. GAPDH was used as the internal reference. Gel Doc EZ Imager (Bio‐Rad, California, USA) was applied for development, and the grey values of target bands were analysed by Image J software. The experiment was repeated three times and the data were averaged.

### 2.17 Dual‐luciferase reporter gene assay

The binding site of miR‐214 and MEG3 or TXNIP was predicted by https://cm.jefferson.edu/rna22/Precomputed. The wild type (WT) MEG3, mutant type (MUT) MEG3, WT TXNIP and MUT TXNIP were constructed. The target fragment was inserted into the pGL3‐control luciferase reporter vectors (Promega, WI, USA) by a restriction endonuclease. Then the luciferase reporter plasmids were independently cotransfected with miR‐NC or miR‐214 into osteoblasts. After 48 hours, cells were lysed and centrifuged at 5000 x g. The luciferase activity was measured with luciferase assay kit (Promega). Renilla luciferase/Firefly luciferase = relative luciferase.

### 2.18 RNA‐pull down assay

Three different biotin‐labelled miRNA sequences Bio‐miR‐214‐WT, Bio‐miR‐214‐MUT and Bio‐NC were designed and synthetized. The osteoblasts were transfected with the above three sequences at 80%‐90% cell confluence. After 48 hours, protein cleavage products were obtained by lysing cells with lysis buffer. Then the lysate was incubated with streptavidin‐coated magnetic beads (M‐280, Sigma‐Aldrich, St. Louis, MO, USA). Finally, the protein‐nucleic acid compound was eluted, and the total RNA was extracted with Trizol, with MEG3 expression detected by RT‐qPCR. Each experiment was repeated three times.

### 2.19 Statistical analysis

Data were analysed with SPSS 21.0 (IBM Corp., Armonk, NY, USA). The measurement data were expressed as mean ± standard deviation. The data between two groups were compared by t test, and those among multiple groups were analysed by one‐way analysis of variance (ANOVA), after which pairwise comparison was performed by the Tukey's post hoc test. *P* was a two‐sided test, and the difference was statistically significant at *P* < 0.05.

## 3 RESULTS

### 3.1 MEG3 and TXNIP are highly expressed while miR‐214 is lowly expressed in femoral tissues of OP rats

To clarify the effect of MEG3/miR‐214/TXNIP axis on the proliferation, differentiation and OPG expression of osteoblasts in OP, MEG3, miR‐214 and TXNIP expression of rat femoral tissues were detected by RT‐qPCR and Western blot analysis (Figure 2A‐E). The results showed that MEG3 and TXNIP expression were pronouncedly enhanced while miR‐214 expression was largely lowered in femoral tissues of OP rats. Subsequently, MEG3 and miR‐214 expression were interfered by si‐MEG3, miR‐214 mimic, OE‐MEG3 + miR‐214 mimic or their NCs, after which MEG3, miR‐214 and TXNIP expression in rats were examined. It was mirrored that MEG3 and TXNIP expression were clearly reduced while miR‐214 expression was obviously augmented by down‐regulating MEG3. In response to miR‐214 mimic treatment, MEG3 expression suggested almost no changes, TXNIP was evidently down‐regulated while miR‐214 was markedly up‐regulated. On the basis of OE‐MEG3 treatment, further treatment of miR‐214 mimic made no change in MEG3 expression, but reduced TXNIP expression and elevated miR‐214 expression. It was indicative that MEG3 and TXNIP were up‐regulated and miR‐214 was down‐regulated in femoral tissues of OP rats and MEG3.

**Figure 2:** MEG3 and TXNIP are up‐regulated while miR‐214 is down‐regulated in femoral tissues of OP rats. A, Detection of MEG3 expression of rat femoral tissues in each group by RT‐qPCR; B, Detection of miR‐214 expression of rat femoral tissues in each group by RT‐qPCR; C, Detection of TXNIP mRNA expression of rat femoral tissues in each group by RT‐qPCR; D, Protein bands of TXNIP of rat femoral tissues in each group; E, Detection of TXNIP protein expression of rat femoral tissues in each group by Western blot analysis; Data were expressed as mean ± standard deviation (n = 10); a, *P* < 0.05 vs the sham group; b, *P* < 0.05 vs the si‐NC group; c, *P* < 0.05 vs the mimic NC group; d, *P* < 0.05 vs the OE‐MEG3 + mimic NC group; data among multiple groups were analysed by ANOVA, after which pairwise comparison was performed by Tukey's post hoc test

### 3.2 MEG3 silencing and miR‐214 overexpression enhance BMD, BV/TV, Tb.N and Tb.Th of femoral tissues in OP rats

Next, the effects of MEG3/miR‐214/TXNIP axis on various indices of rat femoral tissues were investigated. The results indicated that BMD, BV/TV, Tb.N and Tb.Th suggested a reduction in femoral tissues of OP rats. A palpable rise of those indices was achieved by si‐MEG3 or miR‐214 mimic treatment. Although OE‐MEG3 could reduce BMD, BV/TV, Tb.N and Tb.Th levels, rats who subsequently treated with miR‐214 mimic were manifested with increased BMD, BV/TV, Tb.N and Tb.Th values (Figure 3A‐D). It made it comprehensive that MEG3 silencing and miR‐214 overexpression improved BMD, BV/TV, Tb.N and Tb.Th in femoral tissues of OP rats.

**Figure 3:** MEG3 silencing and miR‐214 overexpression enhance BMD, BV/TV, Tb.N and Tb.Th of femoral tissues in OP rats. A, Comparison of BMD in rat femoral tissues in each group; B, Comparison of BV/BT in rat femoral tissues in each group; C, Comparison of Tb.N in rat femoral tissues in each group; D, Comparison of Tb. Th in rat femoral tissues in each group; data were expressed as mean ± standard deviation (n = 10); a, *P* < 0.05 vs the sham group; b, *P* < 0.05 vs the si‐NC group; c, *P* < 0.05 vs the mimic NC group; d, *P* < 0.05 vs the OE‐MEG3 + mimic NC group; data among multiple groups were analysed by ANOVA, after which pairwise comparison was performed by Tukey's post hoc test

### 3.3 MEG3 silencing and miR‐214 overexpression elevate Ca and P contents and reduce ALP content in serum of OP rats

Subsequently, the contents of serum Ca, P and ALP rat serum were detected by the automatic biochemical analyser (Figure 4A‐C). The findings revealed that serum Ca and P contents suggested a decrease while serum ALP content showed a rise in OP rats. MEG3 down‐regulation or miR‐214 up‐regulation elevated serum Ca and P contents while decreased serum ALP content. Moreover, miR‐214 overexpression rescued the effects of MEG3 up‐regulation on serum Ca and P content suppression and serum ALP content promotion in OP rats. It was noticed that MEG3 silencing and miR‐214 overexpression attenuated Ca, P and ALP contents in OP rats.

**Figure 4:** MEG3 silencing and miR‐214 overexpression elevate Ca and P contents and reduce ALP content in serum of OP rats. A, Comparison of Ca content in serum of rats in each group; B, Comparison of P content in serum of rats in each group; C, Comparison of ALP content in serum of rats in each group; data were expressed as mean ± standard deviation (n = 10); a, *P* < 0.05 vs the sham group; b, *P* < 0.05 vs the si‐NC group; c, *P* < 0.05 vs the mimic NC group; d, *P* < 0.05 vs the OE‐MEG3 + mimic NC group; data among multiple groups were analysed by ANOVA, after which pairwise comparison was performed by Tukey's post hoc test

### 3.4 MEG3 silencing and miR‐214 overexpression increase the trabecular bone area and collagen area of femoral tissues in OP rats

To further explore the effects of MEG3/miR‐214/TXNIP axis on rats with OP, the pathological condition of femoral tissues was observed through HE staining and Masson staining (Figure 5A,B). Trabecular bone area and collagen area in rat femurs suggested a distinct reduction in OP rats. Depleting MEG3 or restoring miR‐214 widened trabecular bone area and collagen area. miR‐214 overexpression mitigated the inhibitory role of MEG3 up‐regulation on trabecular bone area and collagen area. It was recognized that silencing MEG3 or overexpression of miR‐214 improved the pathological damage of femoral tissues in OP rats.

**Figure 5:** MEG3 silencing and miR‐214 overexpression increase trabecular bone area and collagen area of femoral tissues in OP rats. A, HE staining of femurs; B, Masson staining of femurs

### 3.5 MEG3 silencing and miR‐214 overexpression up‐regulate OPG protein expression and down‐regulate RANKL protein expression of femoral tissues in OP rats

Next, the potential mechanism of MEG3/miR‐214/TXNIP axis regulating OP was explored. Immunohistochemical staining and Western blot analysis were performed to detect OPG and RANKL protein expression in rat femoral tissues (Figure 6A‐C). The results revealed that OPG protein expression showed a reduction while RANKL protein expression suggested an increase, and OPG/RANKL ratio indicated a decrease in femoral tissues of OP rats. Both si‐MEG3 and miR‐214 mimic could elevate OPG protein expression, lessen RANKL protein expression and increase OPG/RANKL ratio. The impacts of MEG3 overexpression on OPG and RANKL protein expression could be reversed by miR‐214 up‐regulation. It was hinted that MEG3/miR‐214/TXNIP axis affected OPG and RANKL protein expression in rats with OP.

**Figure 6:** MEG3 silencing and miR‐214 overexpression up‐regulate OPG protein expression and down‐regulate RANKL protein expression of femoral tissues in OP rats. A, Detection of OPG and RANKL protein expression in rat femoral tissues by immunohistochemical staining; B, Protein bands of OPG and RANKL in rat femoral tissues by Western blot analysis; C, Comparison of OPG/RANKL values of rat femoral tissues in each group; data were expressed as mean ± standard deviation (n = 10); a, *P* < 0.05 vs the sham group; b, *P* < 0.05 vs the si‐NC group; c, *P* < 0.05 vs the mimic NC group; d, *P* < 0.05 vs the OE‐MEG3 + mimic NC group; data among multiple groups were analysed by ANOVA, after which pairwise comparison was performed by Tukey's post hoc test

### 3.6 Results of osteoblast isolation

Then, the effects of MEG3/miR214/TXNIP axis on OP were clarified through in vitro experiments. Under the inverted microscope, on the 3rd day after the isolation and culture, the cells climbed out of the femoral tissues and were in the shape of short spindle (Figure 7A). The primary cells crawling out merged into a single layer after detachment and were then passaged. The cells attached to the culture dish within 2 to 4 hours and most showed polygonal, shortly fusiform and cuboid shapes. When spreading over the bottom of the bottle, the cells were in fusiform or cuboid shapes and were closely arranged. As the culture time was prolonged, the cells grew in an overlapping and colony‐like manner (Figure 7B). The cells were then identified by VanGieson picric acid‐acid fuchsin staining, ALP staining and ARS staining. The results showed cells were stained brownish red in the VanGieson picric acid‐acid fuchsin staining, indicating that cells had the function of synthesizing matrix proteins (Figure 7C); there were black particles in the cytoplasm, and a few dispersed around the cells, indicating that the ALP activity of cells improved and the cell bone matrix was matured (Figure 7D). When the cells were confluent, they were stacked in multiple layers and showed the shape of short column or square; the cells were aggregated locally to form focus and calcified nodules and showed orange‐red particles or massive precipitates after staining (Figure 7E). It proved that osteoblasts were successfully isolated.

**Figure 7:** Results of osteoblast isolation. A, Observation of osteoblasts climbing out of the femoral tissues 3 d after adherence by the inverted microscope; B, Observation of osteoblasts climbing out of the femoral tissues 7 d after adherence by the inverted microscope; C, VanGieson picric acid‐acid fuchsin staining result; D. ALP staining result; E. ARS staining result

### 3.7 MEG3 silencing and miR‐214 overexpression strengthen osteoblast viability

PCNA and cyclin D1 protein expression of osteoblasts were detected by Western blot analysis (Figure 8A,B), and osteoblast viability was detected by MTT assay (Figure 8C). The results showed that PCNA and cyclin D1 protein expression were down‐regulated and osteoblast viability was weakened in osteoporotic osteoblasts, which would be strengthened by depleting MEG3 or elevating miR‐214. Up‐regulating miR‐214 offset the repression of overexpressed MEG3 on osteoporotic osteoblasts. It was evident that osteoblast proliferation and PCNA and cyclin D1 protein expression were regulated by MEG3/miR‐214/TXNIP axis.

**Figure 8:** MEG3 silencing and miR‐214 overexpression strengthen osteoblast viability. A, Protein bands of PCNA and cyclin D1 in each group; B, Comparison of PCNA and cyclin D1 protein contents in each group by Western blot assay; C, Comparison of OD values in each group; data were expressed as mean ± standard deviation (N = 3); a, *P* < 0.05 vs the sham group; b, *P* < 0.05 vs the si‐NC group; c, *P* < 0.05 vs the mimic NC group; d, *P* < 0.05 vs the OE‐MEG3 + mimic NC group; data among multiple groups were analysed by ANOVA, after which pairwise comparison was performed by Tukey's post hoc test

### 3.8 MEG3 silencing and miR‐214 overexpression enhance COL‐I and COL‐Χ expression and decrease COLII expression of osteoblasts

RT‐qPCR was adopted to detect COL‐I, COL‐II and COL‐Χ expression of osteoblasts (Figure 9A‐C). The results revealed that COL‐I and COL‐Χ expression showed diminution while COL‐II expression suggested enhancement in osteoporotic osteoblasts. Both MEG3 down‐regulation and miR‐214 up‐regulation increased COL‐I and COL‐Χ expression while reduced COL‐II expression. miR‐214 overexpression mitigated the MEG3 up‐regulation‐induced effects on those factors, suggesting that COL‐I, COL‐II and COL‐Χ expression were mediated by MEG3/miR‐214/TXNIP axis.

**Figure 9:** MEG3 silencing and miR‐214 overexpression enhance COL‐I and COL‐Χ expression and decrease COL‐II expression of osteoblasts. A‐C, RT‐qPCR detection of COL‐I, COL‐II and COL‐Χ expression in each group; Data were expressed as mean ± standard deviation (N = 3); a, *P* < 0.05 vs the control group; b, *P* < 0.05 vs the si‐NC group; c, *P* < 0.05 vs the mimic NC group; d, *P* < 0.05 vs the OE‐MEG3 + mimic NC group; data among multiple groups were analysed by ANOVA, after which pairwise comparison was performed by Tukey's post hoc test

### 3.9 MEG3 silencing and miR‐214 overexpression improve osteoblast differentiation ability

OCN, RUNX2 and Osteolix protein expression of rat osteoblasts were detected by Western blot analysis (Figure 10A,B); ALP staining with BCIP/NBT kits was used to qualitatively and quantitatively analyse osteoblast ALP content and activity, and ARS staining to detect mineralized nodule area of osteoblasts (Figure 10C‐E). The results suggested that OCN, RUNX2 and Osteolix protein expression, ALP content and activity and mineralized nodule area of rat osteoblasts were diminished in osteoporotic osteoblasts, indicating decreased osteoblast differentiation ability. Those parameters were enhanced by down‐regulating MEG3 or up‐regulating miR‐214. miR‐214 up‐regulation reversed the function of MEG3 overexpression on those indices. The findings implied that osteoblast differentiation was modulated by MEG3/miR‐214/TXNIP axis.

**Figure 10:** MEG3 silencing and miR‐214 overexpression improve osteoblast differentiation ability. A, Protein bands of OCN, RUNX2 and Osteolix of rat osteoblasts in each group; B, Comparison of OCN, RUNX2, and Osteolix protein expression of rat osteoblasts in each group by Western blot assay; C, Representative results of ALP staining with BCIP/NBT kit and alizarin red staining; D, Comparison of ALP activity of rat osteoblasts in each group; E, Comparison of mineralized nodule area of rat osteoblasts in each group; Data were expressed as mean ± standard deviation (N = 3); a, *P* < 0.05 vs the sham group; b, *P* < 0.05 vs the si‐NC group; c, *P* < 0.05 vs the mimic NC group; d, *P* < 0.05 vs the OE‐MEG3 + mimic NC group; data among multiple groups were analysed by ANOVA, after which pairwise comparison was performed by Tukey's post hoc test

### 3.10 MEG3 specifically binds to miR‐214

To explore whether MEG3 and miR‐214 had a targeting relationship, bioinformatics software https://cm.jefferson.edu/rna22/Precomputed was adopted to predict the specific binding region of MEG3 to the miR‐214 sequence (Figure 11A). The results from further confirmation by dual‐luciferase reporter gene assay revealed that miR‐214 mimic lowered the luciferase activity of the MEG3‐WT, indicating a binding relationship between MEG3 and miR‐214 (Figure 11B). Then, RNA‐pull down assay further verified the relation between MEG3 and miR‐214, as the results revealing that MEG3 expression was increased in Bio‐miR‐214‐WT (Figure 11C).

**Figure 11:** MEG3 specifically binds to miR‐214. A, Bioinformatics software https://cm.jefferson.edu/rna22/Precomputed predicted the binding site between MEG3 and miR‐214 by the bioinformatics software; B, Verification of the regulatory relationship between MEG3 and miR‐214 by dual‐luciferase reporter gene assay; C, Verification of the binding relationship of MEG3 and miR‐214 in osteoblasts by RNA‐pull down assay to; D, MEG3 and miR‐214 expression of osteoblasts in each group; Data were expressed as mean ± standard deviation (N = 3); a, *P* < 0.05 vs the sham group; b, *P* < 0.05 vs the si‐NC group; c, *P* < 0.05 vs the mimic NC group; d, *P* < 0.05 vs the OE‐MEG3 + mimic NC group; e, *P* < 0.05 vs the Inhibitor NC group; data between two groups were compared by t test, and those among multiple groups by ANOVA, after which pairwise comparison was performed by Tukey's post hoc test

We also conducted RT‐qPCR to determine MEG3 and miR‐214 expression (Figure 11D). The results indicated that MEG3 expression increased while miR‐214 expression decreased in osteoblasts of OP rats. MEG3 expression decreased while miR‐214 expression elevated after si‐MEG3 treatment. miR‐214 mimic/inhibitor had no impact on MEG3 expression while elevated/repressed miR‐214 expression. miR‐214 mimic treatment on the basis of OE‐MEG3 enhanced miR‐214 expression but not affected MEG3 expression. It was concluded that MEG3 could competitively bind to miR‐214.

### 3.11 MiR‐214 targets TXNIP

The downstream target genes of miR‐214 were searched. The binding site between TXNIP and miR‐214 was predicted at https://cm.jefferson.edu/rna22/Precomputed (Figure 12A), and dual‐luciferase reporter gene assay was adopted to verify the targeting relation between TXNIP and miR‐214. The results showed that miR‐214 mimic decreased the luciferase activity of TXNIP WT in osteoblasts (Figure 12B), indicating miR‐214 specifically binds to TXNIP.

**Figure 12:** MiR‐214 targets TXNIP. A, Bioinformatics software https://cm.jefferson.edu/rna22/Precomputed prediction of binding site between TXNIP and miR‐214; B, Verification of the regulatory relationship between miR‐214 and TXNIP by dual‐luciferase reporter gene assay; C, Comparison of TXNIP mRNA expression of osteoblasts in each group; D, Protein bands of TXNIP in osteoblasts of each group; E, Comparison of TXNIP protein content of osteoblasts in each group by Western blot assay; data were expressed as mean ± standard deviation (N = 3); a, *P* < 0.05 vs the sham group; b, *P* < 0.05 vs the si‐NC group; c, *P* < 0.05 vs the mimic NC group; d, *P* < 0.05 vs the OE‐MEG3 + mimic NC group; data between two groups were compared by t test, and those among multiple groups by ANOVA, after which pairwise comparison was performed by Tukey's post hoc test

TXNIP expression of transfected osteoblasts was detected by RT‐qPCR and Western blot analysis (Figure 12C‐E). The results showed that TXNIP expression increased in osteoblasts of OP rats, which was reduced by down‐regulating MEG3 or enhancing miR‐214. miR‐214 inhibition caused a decrease in miR‐214 expression and an increase in TXNIP expression. Also, miR‐214 up‐regulation reversed the promoting effect of MEG3 overexpression on TXNIP expression. It was summarized that TXNIP was targeted by miR‐214 and mediated by MEG3/miR‐214 axis.

## 4 DISCUSSION

OP, a ubiquitous public health problem (especially in women), is characterized by reduced bone strength which is easy to lead to an incremental risk for fracture.^15^ Recently, lncRNAs have been confirmed as a novel regulatory code for OP.^16^ Here, we discussed the mechanism of lncRNA MEG3 on OP via modulating miR‐214 and TXNIP. Collectively, we demonstrate that knockdown of MEG3 and elevation of miR‐214 enhance OPG expression, and boost proliferation and differentiation of osteoblasts in OP by down‐regulating TXNIP, which further improves OP (Figure 13).

**Figure 13:** The mechanism of MEG3/miR‐214/TXNIP axis in osteoblast differentiation. LncRNA MEG3 regulates osteoblast differentiation through miR‐214/TXNIP axis to modulate OPG/RANKL ratio

To start with, we conducted assays to found that lncRNA MEG3 and TXNIP were higly expressed while miR‐214 was lowly expressed in femoral tissues of OP rats. Similar to our results, a recent study has showed that MEG3 is up‐regulated in postmenopausal OP.^6^ Another study by Cai N *et al* have proposed that lncRNA ANCR expression is also augmented in postmenopausal OP.^17^ There has been evidence proving that miR‐214 expression is low in some disease, such as ovarian cancer and breast cancer.^18^, ^19^ In a previous study, Lekva T *et al* have reported the high TXNIP mRNA level in Cushing's syndrome.^20^ TXNIP has also been documented to be overexpressed in hepatocyte ischaemia reperfusion injury.^21^ What's more, we also discovered that MEG3 specifically bound to miR‐214 to modulate TXNIP expression, and reduced MEG3 expression caused a rise in miR‐214 expression which could declined TXNIP expression. Studies have shown that MEG3 works as a ceRNA of miR‐214 and decreased MEG3 expression augments miR‐214 expression.^22^ It has also been indicated that TXNIP is miR‐224’ target and miR‐224 negatively modulates TXNIP expression.^23^

To better figure out the mechanism of lncRNA MEG3 on OP development, si‐MEG3 and miR‐214 mimic were introduced into assays performed in femoral tissues in OP rats and osteoblasts. We found that MEG3 silencing and miR‐214 overexpression increased BMD, BV/TV, Tb.N, Tb.Th, the number of osteoblasts, collagen area and OPG expression and down‐regulated RANKL of femoral tissues in OP rats. What was also discovered in our study was that MEG3 silencing and miR‐214 overexpression elevated Ca and P contents and reduced ALP content in OP rats’ blood, elevated viability, differentiation ability, COL‐I and COL‐Χ contents and ALP activity, and abated COL‐II content of osteoblasts. In addition, we combined OE‐MEG3 and miR‐214 mimic in our assays, and found that miR‐214 restoration counteracts the effects of MEG3 up‐regulation on OP and osteoblasts. As proved, MEG3 has been revealed to induce hepatic insulin resistance via sponging miR‐214.^22^ Moreover, MEG3 and miR‐214 functioned in combination to regulate the growth of T‐cell lymphoblastic lymphoma cells.^7^ As discussed previously, MEG3 is involved in osteogenic differentiation of multiple MSCs and crucially mediates the development of bone formation and associated diseases.^24^ Moreover, MEG3 inhibition could suppress the activation of bone morphogenetic protein 4 signalling and then contributes to osteogenic differentiation in OP.^25^ In line with our results, a recent report has revealed that MEG3 silencing increases the levels of COL10A1, Runx2, Osterix and OCN, which speeds up tibia fraction healing.^26^ Evidence has shown that lncRNA ANCR silencing enhances the proliferation, calcium deposition and ALP activity and diminished apoptosis of osteoblasts, which facilitates the osteogenesis of osteoblast in postmenopausal OP by modulating EZH2 and RUNX2.^17^ Some researchers have also proffered that diminution of MEG3 catalyzes endothelial differentiation of BMSCs in restoring erectile dysfunction.^27^ In addition, Wang Y *et al* have demonstrated that MEG3 knockdown limits osteosarcoma cell development via modulating miR‐127.^28^ A prior study has suggested that lncRNA MEG3 up‐regulation dampens the osteogenic differentiation of periodontal ligament cells.^29^ It has been shown that restoration of miR‐214 contributes to osteoclast differentiation.^30^ Beside, there has been literature recording that in cervical cancer, miR‐214 controls cancer cell growth and invasion by down‐regulating ARL2.^31^ Furthermore, miR‐214 increases breast cancer cell apoptosis and sensitivity to doxorubicin via modulating the RFWD2‐p53 cascade.^32^

All in all, we reveal that knockdown of MEG3 and elevation of miR‐214 strengthen OPG expression, and boost proliferation and differentiation of osteoblasts in OP by down‐regulating TXNIP, thus mitigating OP. Our study promotes better understanding of the function of MEG3/miR‐214/TXNIP axis in OP development and provides new clues for OP treatment. However, in‐depth research has to be made to further elaborate the mechanism of lncRNA MEG3 on OP development.

## FUNDING

Project supported by the Natural Science Foundation of Guangdong Province, China (Grant No.2020A151501711).

## CONFLICT OF INTEREST

The authors declare that they have no conflicts of interest.

## AUTHOR CONTRIBUTION

**Rui Ding:** Writing‐original draft (equal). **ZhengTao Gu:** Data curation (equal). **ChangSheng Yang:** Formal analysis (equal). **CaiQiang Huang:** Formal analysis (equal). **QingChu Li:** Data curation (equal). **DengHui Xie:** Formal analysis (equal). **RongKai Zhang:** Formal analysis (equal). **YiYan Qiu:** Writing‐original draft (equal).
